The article "Regression Analysis of Factors Based on Cluster Analysis of Acute Radiation Pneumonia due to Radiation Therapy for Lung Cancer" was retracted in 2023. Reasons: signs of a paper mill; suspected computer-generated content; unreliable results or conclusions; lack of ethics approval or compliance.

# Regression Analysis of Factors Based on Cluster Analysis of Acute Radiation Pneumonia due to Radiation Therapy for Lung Cancer

**DOI:** 10.1155/2021/3727794

**Published:** 2021-10-13

**Authors:** Xiaofeng Zhang, Beili Lv, Lijun Rui, Liming Cai, Fenglan Liu

**Affiliations:** ^1^Respiratory Department, The Affiliated Hospital of Jiangnan University, Wuxi Jiangsu 214062, China; ^2^Medical School Liaocheng University, Shandong Liaocheng 250200, China

## Abstract

We conducted in this paper a regression analysis of factors associated with acute radiation pneumonia due to radiation therapy for lung cancer utilizing cluster analysis to explore the predictive effects of clinical and dosimetry factors on grade ≥2 radiation pneumonia due to radiation therapy for lung cancer and to further refine the effect of the ratio of the volume of the primary foci to the volume of the lung lobes in which they are located on radiation pneumonia, to refine the factors that are clinically effective in predicting the occurrence of grade ≥2 radiation pneumonia. This will provide a basis for better guiding lung cancer radiation therapy, reducing the occurrence of grade ≥2 radiation pneumonia, and improving the safety of radiotherapy. Based on the characteristics of the selected surveillance data, the experimental simulation of the factors of acute radiation pneumonia due to lung cancer radiation therapy was performed based on three signal detection methods using fuzzy mean clustering algorithm with drug names as the target and adverse drug reactions as the characteristics, and the drugs were classified into three categories. The method was then designed and used to determine the classification correctness evaluation function as the best signal detection method. The factor classification and risk feature identification of acute radiation pneumonia due to radiation therapy for lung cancer based on ADR were achieved by using cluster analysis and feature extraction techniques, which provided a referenceable method for establishing the factor classification mechanism of acute radiation pneumonia due to radiation therapy for lung cancer and a new idea for reuse of ADR surveillance report data resources.

## 1. Introduction

Lung cancer, also known as primary bronchopulmonary cancer, is a malignant tumour that occurs mainly in bronchial mucosal epithelial cells, with a few occurring in alveolar tissue. Patients with lung cancer often have no obvious clinical symptoms in the early stage of the disease and are often neglected. As the disease worsens and develops to the middle and late stage, they start to show clinical symptoms such as haemoptysis and pain. Most of the patients have already developed to the middle and late stages when their disease is discovered, and the best time for surgical treatment is lost [1]. The diagnosis of lung cancer is relatively easy. Combining clinical symptoms, imaging (CT, MRI, etc.), and biochemical indexes can make a preliminary diagnosis of the patient's disease status, and for patients suspected of having lung cancer, the pathological examination can make a definite diagnosis. Radiotherapy is one of the main treatment methods for lung cancer, and clinical statistics show that more than 70% of lung cancer patients need radiotherapy during treatment, indicating the important value of radiotherapy in lung cancer treatment [2]. For measurement data, independent-sample *t*-test or nonparametric rank-sum test is used in multivariate analysis of variance. The main treatment mechanism of radiotherapy is to irradiate tumour tissues and cells with high doses of radiation to kill cancer cells and prevent their continued proliferation and differentiation [3]. However, during radiotherapy, a large area of noncancerous lung tissue will be exposed to radiotherapy, normal lung tissues do not have good tolerance to high-dose radiation, and the normal lung tissues will be damaged to different degrees under high-dose radiation. The lung tissue damage caused by radiotherapy is a kind of value-added death damage. After high-dose radiation irradiation, cell damage immediately appears and a series of cytokine synthesis increases, which triggers a series of pathophysiological reactions with the transmission and amplification of intercellular signals, thus causing radiation pneumonia. The occurrence of radiation pneumonia not only affects the normal effect of radiotherapy but also has a serious impact on the patient's recovery, leading to a decrease in the patient's quality of life.

The article "Regression Analysis of Factors Based on Cluster Analysis of Acute Radiation Pneumonia due to Radiation Therapy for Lung Cancer" was retracted in 2023. Reasons: signs of a paper mill; suspected computer-generated content; unreliable results or conclusions; lack of ethics approval or compliance.

The main goal of cluster analysis is to divide the samples or feature variables into a data set by distance so that the distance between elements in the same class is closer than the distance between elements in other classes, or the elements in the same class are more similar than other classes so that the homogeneity of elements within classes and the heterogeneity of elements between classes can be maximized at the same time [2]. Image cutting uses the Image Segmented tool software in the MATLAB software, using a semiautomatic method. After the approximate range is manually outlined, the software automatically iteratively calculates. A good clustering model can solve the problem of large data size [4]. Cluster analysis divides the given data by its inherent characteristics, to better grasp the data characteristics of each cluster after the division, reduce the size of the data, and obtain simpler and more intuitive data from the relatively complex original data. It is also possible to obtain simpler and more intuitive data from the relatively complex original data and uncover the hidden data value behind the huge data volume. Therefore, cluster analysis has become a very important part of big data analysis, and it has been successfully applied to many practical problems in social and natural sciences. For example, in the financial industry, cluster analysis can be used for bank customer segmentation and financial investment; in traffic management, cluster analysis can be used for traffic control and traffic accident analysis; in the biomedical field, cluster analysis can study the nature and function of genes and proteins, thus helping us to explore the mystery of life.

At present, the incidence of acute radiation pneumonia after radiotherapy for lung cancer patients is relatively high, which not only affects the effect of radiotherapy but also increases the incidence of complications and increases the risk of radiotherapy. Taking reasonable measures to reduce the incidence of acute radiation pneumonia after radiotherapy for lung cancer patients is an important research topic for clinical workers, which becomes a major clinical complication. The occurrence of acute radiation pneumonia will hinder normal treatment, leading to the inability to increase the radiation dose, the clinical treatment effect is very poor, and the patient's quality of life is not ideal. This study aims to investigate the risk factors associated with acute radiation pneumonia in lung cancer patients after radiotherapy and to guide clinicians to take reasonable treatment measures to prevent the occurrence of acute radiation pneumonia according to the actual situation of patients, to improve the clinical effect of lung cancer radiotherapy and reduce the risk of radiation pneumonia. It is important to improve the clinical effect of radiotherapy and reduce the occurrence of complications.

## 2. Related Work

Many clinical factors have been reported to influence the development of radiation pneumonia, including age, gender, smoking history, and history of chronic obstructive pulmonary disease (COPD). Wang et al. reported that age was an influential factor in the development of radiation pneumonia and that patients of advanced age were at a higher risk of developing radiation pneumonia [5]. Tinkle et al. showed that smoking history was a protective factor against radiation pneumonia and that smoking could prevent radiation pneumonia [3]. The risk and severity of radiation pneumonia are higher in patients with a history of severe COPD [6]. The effect of concurrent radiotherapy on the occurrence of radiation pneumonia has been inconsistently concluded in different studies, which mainly lies in the different toxic effects on lung tissues by using different chemotherapeutic drugs [7]. Many drugs for oncology cause an increased risk of developing radiation pneumonia, such as methotrexate, bleomycin, and mitomycin, which have pulmonary toxicity and can increase the risk of radiation pneumonia [8]. There is no solid evidence to support the fact that classical oncology chemotherapy drugs such as cisplatin and carboplatin increase the risk of radiation pneumonia. However, more chemotherapeutic agents such as paclitaxel and gemcitabine show greater pulmonary toxicity in concurrent radiotherapy sensitization therapy, which can lead to an increased risk of radiation pneumonia. Therefore, try to avoid the use of these drugs with pulmonary toxicity during radiotherapy to reduce the risk of radiation pneumonia.

The article "Regression Analysis of Factors Based on Cluster Analysis of Acute Radiation Pneumonia due to Radiation Therapy for Lung Cancer" was retracted in 2023. Reasons: signs of a paper mill; suspected computer-generated content; unreliable results or conclusions; lack of ethics approval or compliance.

Among the many dosimetry parameter studies reported so far, dosimetry parameters such as V5, V20, and V30 have the greatest value in predicting the risk of radiation pneumonia and are now used in clinical practice to improve the ability to predict the risk of radiation pneumonia, but Pradhan et al. reported in a review study of current clinically applied dosimetry assessment parameters that, even at lower dosimetry reference values, radiation pneumonia still occurs, and it is not yet possible to accurately predict the occurrence of radiation pneumonia [9]. In clinical practice, we observed that, with the increase of radiotherapy dose, the radiation dose and irradiation volume of the lung lobe of the primary focus were higher than those of the adjacent lobe and the chance of radiation pneumonia in the lung lobe of the primary focus was higher than that of the adjacent lobe [10]. There are few reports in the domestic and international literature about the relationship between the volumetric dosimetry of radiation and radiation pneumonia in the lung lobe where the primary focus of lung cancer is located; therefore, this topic will explore the clinical factors and dosimetry factors on radiotherapy-induced radiation pneumonia in lung cancer [11]. Therefore, this study will investigate the predictive role of clinical and dosimetry factors on the development of ≥2-grade radiation pneumonia due to lung cancer radiotherapy and refine the effect of the ratio of the volume of the primary foci to the volume of the lung lobes in which they are located on ≥2-grade radiation pneumonia, to refine the factors that are clinically effective in predicting the development of ≥2-grade radiation pneumonia and provide a basis for better guiding lung cancer radiotherapy, reducing the risk of ≥2-grade radiation pneumonia, and improving the safety of radiotherapy [12]. It has been pointed out that many factors are leading to acute radiation pneumonia in lung cancer radiotherapy patients, including patients' clinical factors, physical factors of radiotherapy, and biological factors. However, at this stage, the research on factors related to acute radiation pneumonia in lung cancer patients after radiotherapy lacks systematicity and cannot provide good scientific guidance for clinical prevention.

The article "Regression Analysis of Factors Based on Cluster Analysis of Acute Radiation Pneumonia due to Radiation Therapy for Lung Cancer" was retracted in 2023. Reasons: signs of a paper mill; suspected computer-generated content; unreliable results or conclusions; lack of ethics approval or compliance.

The BIRCH algorithm uses clustering features and CF trees instead of cluster descriptions, thus achieving efficiency and scalability in large datasets, making the method suitable for incremental and dynamic clustering. On the other hand, it is based on the idea of representative points, which is a good solution to the problem of clustering preference for spherical shapes and similar cluster sizes and is also more robust in dealing with isolated points. And to solve the problem that the divisional clustering method cannot effectively deal with complex-shaped datasets, a density-based clustering algorithm DBSCAN algorithm was proposed, which does not use the conventional method of measuring data similarity by distance but divides the dataset by sparsity of density, and such an approach can discover clusters of various shapes in complex datasets with noise. With the development of clustering algorithms, grid-based and density-based clustering algorithms also emerged later and have been well studied and maturely applied. The classification results of the first two types of flowers are ideal, while the third type of flowers has a higher misjudgement. There is a small overlap between the latter two categories. This may be related to the size of the data. Too small data size causes the clustering algorithm to fail. Learn all kinds of characteristics more effectively. The GA indicator of clustering effectiveness based on generalization ability is proposed, and the method of determining the optimal number of clusters for K-means based on the GA indicator is proposed by combining the indicator with the K-means algorithm. Through experiments, it is proved that the method works well in determining the optimal number of clusters.

## 3. Regression Analysis of Factors for Acute Radiation Pneumonia due to Radiation Therapy for Lung Cancer by Cluster Analyses

### 3.1. Clustering Analysis Algorithm Design

Cluster analysis is a type of unsupervised learning, also known as unguided learning, and a common method in multivariate statistical analysis, which is an important research element in the fields of data mining, machine learning, and pattern recognition [13]. The difference between cluster analysis and supervised learning methods is that the samples used in cluster analysis are not labelled in advance, and the categories to which the samples belong are determined automatically by the cluster analysis algorithm, which is a process of dividing the data set into clusters according to the similarity of the samples' characteristics without training data so that the samples within the same cluster have high similarity and the samples in different clusters have high dissimilarity. Although cluster analysis has a history of several decades, there is no unified definition of cluster analysis so far because different clustering methods end up with a variety of output patterns of the cluster structure. Among the various ways of defining cluster analysis, the one that is accepted by most people is the mathematical description given based on the most common form of output in cluster analysis, the K-split of the sample data.

The article "Regression Analysis of Factors Based on Cluster Analysis of Acute Radiation Pneumonia due to Radiation Therapy for Lung Cancer" was retracted in 2023. Reasons: signs of a paper mill; suspected computer-generated content; unreliable results or conclusions; lack of ethics approval or compliance.

Let the dataset *X*={*x*_1_, *x*_2_, ..., *x*_*n*_} and *R* be the clusters defined on the dataset *X* . Split *X* into *m* set classes *C*_1_, ..., *C*_*m*_ , if these *m* set classes satisfy the following three conditions:

(1) $$\begin{array}{c} C_{i}\neq \phi ,\\ \cup_{i=1}^{m}C_{i}=X,\\ C_{i}\cap C_{j}=\phi . \end{array}$$

Then, it is said to be a cluster on dataset X. Among the above three conditions, condition 1 restricts that all set classes are nonempty, condition 2 restricts that all sample points in dataset *X* have set classes to which they belong, and condition 3 constrains that each set class does not intersect with each other. From these three constraints, it can be summarized that any sample point in dataset *X* will be classified into an ensemble class and can belong to at most one ensemble class [14]. Finally, based on the obtained risk grading results and the signal proportion sum, the pharmacological correlation of each drug category was analysed and evaluated by the drugs of each risk level to further verify the rationality and feasibility of this experiment. Although the diversity of clustering criteria leads to different clustering results obtained by different clustering methods, basically all clustering methods need to follow the following four steps. Preprocess the data and feature engineering to retain as much information as possible in the processed data. The clustering algorithm is selected according to the structure of the data; the validity of the clustering results is checked by selecting the appropriate clustering validity index; the clustering results are analysed together with other experimental data to understand the clustering results; and the final correct conclusion is obtained, as shown in Figure 1.

The article "Regression Analysis of Factors Based on Cluster Analysis of Acute Radiation Pneumonia due to Radiation Therapy for Lung Cancer" was retracted in 2023. Reasons: signs of a paper mill; suspected computer-generated content; unreliable results or conclusions; lack of ethics approval or compliance.

Based on this study, cluster analysis is an exploration of the intrinsic association of adverse reactions to antibiotics, but no specific number of clusters is specified, and the number of clusters needs to be determined artificially for a more stable and reasonable clustering effect. In this study, the elbow rule was used to determine the clustering values [15]. The main idea of the elbow rule is to record and plot the objective function value of each clustering value. As the objective function value increases, the average distortion decreases; each category contains fewer objects accordingly, so the objects will be closer to their centres; however, as the number of clusters increases, the level of change of the average distortion continues to decrease. As the number of clusters increases, the clustering value corresponding to the place where the level of aberration decreases the most is the elbow, and the clustering value corresponding to the elbow can be used as the best clustering value for cluster analysis. To derive the best clustering number more intuitively, this paper proposes to use the method of calculating the angle between two lines, and the absolute value of the tangent of the angle is the best clustering number. The tangent formula for the angle is as follows:

(2) $$\begin{array}{c} EI_{\mathrm{drug}}=\sum_{n=1}^{s}\frac{N_{\mathrm{yn}}}{N_{\mathrm{tn}}}k_{n}^{2}. \end{array}$$

We scored each type of antibiotic based on the severity of adverse reactions. General adverse reaction type was rated as 1 point, and severe adverse reaction type was rated as 3 points. Adverse drug reaction injury index is defined as follows:

(3) $$\begin{array}{c} DI_{\mathrm{ADR}}=\frac{\sum_{n=1}^{s}N_{\mathrm{yn}}/N_{\mathrm{tn}}k_{n}^{2}}{m}, \end{array}$$

where *n* denotes the number of adverse reactions where the reported type of each drug is average, *n* denotes the number of adverse reactions where the reported type of each drug is serious, and *n* denotes the number of drugs in each category [16]. Because of the existence of drugs with a serious number of 0, this study intends to score the adverse reaction impairment index for such drugs as 1. According to the sensitivity and misjudgement rate of the whole lung V20 at each point on the ROC curve, the values of all cut-off points (sensitivity + specificity) are calculated. The diagnostic index corresponding to the maximum cut-off point is that the best diagnostic threshold is 25.9%. In the definition of adverse reaction severity score, the higher the severity of adverse reactions which scored higher, the higher the calculated adverse drug reaction impairment index and the higher the risk level of the corresponding class of drugs.

The article "Regression Analysis of Factors Based on Cluster Analysis of Acute Radiation Pneumonia due to Radiation Therapy for Lung Cancer" was retracted in 2023. Reasons: signs of a paper mill; suspected computer-generated content; unreliable results or conclusions; lack of ethics approval or compliance.

There are three main types of internal validity metrics, namely, metrics based on sample geometry of datasets, metrics based on dataset partitioning, and metrics based on statistical information of datasets. There are many internal validity metrics, including Want metric, CH metric, Hart metric, KL metric, DB metric, and IGP metric. They are more commonly used. Among them, the In-Group Proportion (IGP) indicator is based on the statistical information of the dataset, while all other indicators are based on the structure of the sample set of the dataset. These internal validity indicators are not based on external characteristics as a reference standard, but on the statistical characteristics of the dataset itself to assess the validity of the clustering results, so these clustering validity indicators can be used as the selection criteria for the optimal number of clusters. The idea of the CH indicator is to represent the separation by the class matrix and the tightness by the intraclass deviation matrix.

(4) $$\begin{array}{c} \mathrm{CH}\left(k\right)=\frac{\mathrm{tr}B\left(k\right)/k}{\mathrm{tr}W\left(k\right)/n}. \end{array}$$

Although there are many existing clustering algorithms, most of them need to determine the number of clusters in advance, and the number of clusters as a hyperparameter in the clustering algorithm often has a great influence on the clustering results. In the early days of cluster analysis, the number of clusters was often set artificially by data analysts through experience or by combining background and knowledge from other fields, which was too crude and subjective to obtain the best clustering results. At present, the optimal number of clusters is mostly determined by combining the clustering algorithm with the internal validity index, the internal validity index is used to evaluate the clustering results under different clustering numbers, and the number of classes corresponding to the best clustering validity is selected as the optimal number of clusters for the data set, as shown in Figure 2.

An overview of cluster analysis is given, including the definition of cluster analysis, the basic steps, and the five classes of clustering algorithms. Then the evaluation of cluster validity is introduced, and several classical external validity indicators, as well as internal validity indicators, are presented, respectively. Finally, the method for determining the optimal number of clusters is described in detail, and the algorithmic steps for determining the optimal number of clusters are expressed in the form of an algorithmic flowchart. As the disease worsens, it progresses to the middle and late stages and begins to show clinical symptoms such as haemoptysis and pain. Most patients have already progressed to the middle and late stages when the disease is discovered and have lost the best period of surgical treatment. This chapter introduces the relevant knowledge background to pave the way for the subsequent chapters and provides the theoretical basis for the algorithm simulation experiments in the future.

The article "Regression Analysis of Factors Based on Cluster Analysis of Acute Radiation Pneumonia due to Radiation Therapy for Lung Cancer" was retracted in 2023. Reasons: signs of a paper mill; suspected computer-generated content; unreliable results or conclusions; lack of ethics approval or compliance.

Clustering validity analysis generally refers to the process of evaluating the merit of clustering results. Intuitively, the merit of clustering results lies in the accuracy of the clustering of samples in the dataset, and most of the existing external validity evaluation metrics are proposed for this point. However, in practical applications, the real clustering of samples in the dataset is difficult to obtain, and this limitation makes it difficult to ensure the practicality of external validity metrics. Unlike external validity indexes, internal validity indexes are often used to test whether the clustered dataset can reflect the intrinsic structure of the dataset, that is, whether the dataset can be as similar as possible while the samples between classes are as different as possible after clustering. Therefore, internal validity metrics are mostly based on the idea of the maximum-minimum distance of sample points, and the objective function is to minimize the intraclass distance and maximize the interclass distance in the clustering results.

(5) $$\begin{array}{c} X_{\mathrm{tr}}=\left\{x_{\mathrm{tr}}^{1},x_{\mathrm{tr}}^{2},...,x_{\mathrm{tr}}^{m}\right\}. \end{array}$$

The GA metric evaluates clustering results in terms of generalization ability in guided learning based on the current clustering results; that is, it considers the merit of clustering results to be related to their generalization ability to predict unknown samples and therefore differs from existing clustering validity metrics, whether external or internal. The clustering results of the training set are used for machine learning to build a classifier, and this classifier is used to predict the test set and compare the prediction results with the clustering results. Therefore, GA metrics are like external validity metrics, but the difference is that it is difficult to obtain the true category of the dataset with the commonly used external validity metrics, while GA metrics solve the problem of difficulty in obtaining the true category of the dataset by constructing a classifier and replacing the true category of the test dataset with the predicted result of the classifier.

The article "Regression Analysis of Factors Based on Cluster Analysis of Acute Radiation Pneumonia due to Radiation Therapy for Lung Cancer" was retracted in 2023. Reasons: signs of a paper mill; suspected computer-generated content; unreliable results or conclusions; lack of ethics approval or compliance.

### 3.2. Factor Regression Experiment of Acute Radiation Pneumonia due to Radiation Therapy for Lung Cancer

The relevant medical records of all study subjects were retrieved using the electronic medical record system: general information (gender, age, smoking history, history of chronic lung disease, combined diabetes mellitus, and prechemotherapy FEV1), disease (clinical stage, pathological type, and tumour location), albumin and haemoglobin levels, and relevant treatment (chemotherapy cycle before radiotherapy, whether radiotherapy was applied simultaneously, mean lung dose (MLD), V5, V20, V30, etc.). According to the occurrence of acute radiation pneumonia, the study subjects were divided into the acute radiation pneumonia group and the normal radiotherapy group, and the differences in the indexes between the two groups were compared to analyse the risk factors associated with the development of acute radiation pneumonia after radiotherapy in lung cancer patients [17]. The differences between the two groups in terms of general information, disease, albumin and haemoglobin levels, and related treatment were observed and compared. Patients were followed up for 6 months, and the treatment status of both groups was recorded in detail. Follow-up visits included telephone calls and a review of patients' imaging information. The follow-up included the patients' clinical symptoms and chest CT imaging performance.

The data involved in this study were analysed and processed using SPSS 20.0 statistical software. For the count data, the data were expressed in the form of percentages (%), and the results of comparison between the data were tested using 2, with *P* < 0.05as a statistically significant difference; for the measurement data, the data were expressed using, the results of comparison between the data were tested using *t*, and 0.05 was considered statistically significant. The unconditional logistic regression model was used to analyse the risk factors for acute radiation pneumonia after radiotherapy in lung cancer patients, and the OR values and their confidence intervals (95% CI) were calculated [18]. In the acute radiation pneumonia group, the percentages of patients with lower middle lobe lung cancer, history of chronic lung disease, combined diabetes mellitus, and the percentages of patients with smoking history were significantly lower than those in the normal radiotherapy group. The percentage of patients with a smoking history was significantly lower than that of the normal radiotherapy group, and the comparison was statistically significant. However, there were no significant differences between the two groups in terms of gender, age, clinical stage, pathological type, albumin, and haemoglobin levels, as shown in Figure 3.

The article "Regression Analysis of Factors Based on Cluster Analysis of Acute Radiation Pneumonia due to Radiation Therapy for Lung Cancer" was retracted in 2023. Reasons: signs of a paper mill; suspected computer-generated content; unreliable results or conclusions; lack of ethics approval or compliance.

The diagnosis of radiation pneumonia is mainly exclusionary and must be accompanied by the following conditions: history of previous lung irradiation; chest CT imaging mainly shows patchy images, ventilated bronchial signs, striae, solid lung images, or honeycomb-like changes confined to the radiation field, the lesions do not correspond to the anatomical structure of normal lung tissue (not distributed according to lung fields or lung segments), and a small number of patients in the acute phase of the injury may have imaging changes outside the radiation field in addition to those in the irradiated area. In addition to changes in the irradiated area, a few patients may also have imaging changes outside the radiation field; patients with severe lung injury have clinical symptoms such as cough, shortness of breath, and fever. Cough is the most common, followed by shortness of breath; patients with mild lung injury have shortness of breath after activity; patients with severe lung injury also feel shortness of breath in a calm state; about 50% of patients have a fever; the above symptoms are excluded due to the following factors [19]. Under high-dose radiation, normal lung tissues will be damaged to varying degrees. The above symptoms are excluded from the following factors: tumour progression, lung infection (bacterial, fungal, or viral), acute exacerbation of COPD, cardiogenic disease, pulmonary infarction, anaemia, and drug-related pneumonia.

The first radiation treatment was used as the starting time point, the occurrence of acute radiation pneumonia was recorded within 90 days, and grade 2 radiation pneumonia was used as the endpoint of this study. In the one-way ANOVA, the independent binary chi-square test was chosen for the analysis of count data, and the independent-sample *t*-test or nonparametric rank-sum test was used for the analysis of measurement data; in the multifactor ANOVA, the binary logistic regression analysis was chosen to determine the test level *a* = 0.05, and *P* < 0.05 was taken as statistically significant.

The dose drop rate at the edge of the target area is faster, and to improve the resolution of the dose by the spatial information model, the outward expansion step in the direction of all endangered organs is smaller in the range closer to the target area. Since the dose outside the target area had different dose drop ranges in the bladder, small bowel, rectum, and femoral head directions, the dose drop rate was faster in the rectum and femoral head directions compared to the bladder and small bowel directions, and therefore, their outward expansion steps were smaller relative to the bladder and small bowel directions. All images for texture cut were in 2D mode, and CT image cut was selected by scanning the largest level, measuring the CT value of the lesion and the diameter of the lesion, and then performing image cut. After high-dose radiation exposure, cell damage appears immediately, followed by a series of cytokine synthesis increases. With the transmission and amplification of signals between cells, a series of pathophysiological reactions are triggered, which leads to radiation pneumonitis. The Image Segmented tool within the MATLAB software introduced in the previous chapter was used to perform the image segmentation in a semiautomatic manner, with the approximate extent outlined manually and then iterated automatically by the software, paying attention to the structures adjacent to the chest wall vessels, mediastinum, and atelectasis, as shown in Figure 4.

The article "Regression Analysis of Factors Based on Cluster Analysis of Acute Radiation Pneumonia due to Radiation Therapy for Lung Cancer" was retracted in 2023. Reasons: signs of a paper mill; suspected computer-generated content; unreliable results or conclusions; lack of ethics approval or compliance.

With the increasing level of awareness of radiation pneumonia, people began to pay attention to the risk factors that induce acute radiation pneumonia and tried to take effective measures in clinical treatment to reduce the incidence of acute radiation pneumonia and ensure the clinical treatment effect. Some foreign researchers have taken lung cancer patients receiving radiotherapy as study subjects and formulated radiotherapy regimens for them according to the target population's characteristics, with targeted restrictions on radiotherapy dose and volume, resulting in a significant reduction in the incidence of acute radiation pneumonia [20]. No matter what kind of radiotherapy will inevitably cause damage to good cells and tissues, the incidence of various complications in radiotherapy patients is high, such as hair loss, skin reaction, immunosuppression, bone marrow suppression, nephrotoxicity, pulmonary toxicity, gastrointestinal toxicity, and radiotherapy pneumonia.

In recent years, the incidence of acute radiation pneumonia after radiotherapy treatment for lung cancer patients is high and has become a major complication in clinical practice. The occurrence of acute radiation pneumonia will hinder the normal treatment, resulting in the inability to enhance the radiation therapy dose, poor clinical treatment effect, and unsatisfactory life quality of patients. In severe cases, it may even lead to interruption of treatment and induce death.

## 4. Analysis of Results

### 4.1. Cluster Analysis Results

The data in the original database included the drug classification, drug name, ADR name, the number of reports of both the target drug and the target ADR in the database a value, the total number of all other ADRs for the target drug *b* value, the total number of targets ADRs for drugs other than the target drug in the database *c* value, and the total number of reports other than the target drug and the target ADR in the entire databased value. The corresponding PRR values, IC values, and binary values were calculated by substituting each value into the formula in the previous chapter, and the information obtained is shown in Figure 5.

The article "Regression Analysis of Factors Based on Cluster Analysis of Acute Radiation Pneumonia due to Radiation Therapy for Lung Cancer" was retracted in 2023. Reasons: signs of a paper mill; suspected computer-generated content; unreliable results or conclusions; lack of ethics approval or compliance.

To cluster the drugs, this paper builds a vector space model with the selected drugs and the signal detection values of the adverse reactions as features and outputs the results as a cross-tabulation table. The following is the cross-wizard table generated with the binary value data, IC value data, and PRR value data as features, respectively. The vector space model was established with the antibiotic name as the row label and each type of adverse reaction as the column label, where the binary value of the adverse reaction-antibiotic combination without signal was set as 0. The clustering results were compared with the category to which the original samples belonged, and it was found that 136 samples were accurately classified out of all 150 samples. The classification results were more satisfactory for the first two flowers, while the misclassification was higher for the third flower.

There was a small overlap between the latter two categories, which may be related to the size of the data volume, too small to cause the clustering algorithm to learn the features of each category more effectively, thus leading to misclassification of the clustering results. The basic structure of these three datasets is briefly introduced before the experiment. The BUPA dataset has 345 samples with sample dimension 6 and correct class number 2; the PID dataset has 768 samples with sample dimension 8 and correct class number 2; the BCW dataset consists of 699 samples with sample dimension 9 and correct class number 2.

The data preprocessing process of this risk classification model based on cluster analysis was described in detail. Firstly, the data set and data sources used in this study were introduced, the selected drugs and the WHO adverse drug reaction terminology set used for the query were presented in the form of a list, and then the vector space model was established based on the reported data with three signal detection methods, namely, PRR, IC, and binary value, respectively. In order to select the signal detection methods suitable for cluster analysis, realize the drug risk classification, and verify the credibility of the experimental results, this study firstly screened the common signal detection methods and initially determined three signal detection methods, namely, PRR, IC, and binary value; then the best clustering numbers of the three methods were derived based on the elbow rule, and the best clustering numbers of each method were used to conduct the MATLAB simulation tool. In this way, the homogeneity of the elements within the class and the heterogeneity of the elements between the classes are maximized at the same time. An important feature of the data in the era of big data is the huge amount of data. A good clustering model can just solve the data. The specific results of the clustering of these three signal detection methods were substituted into the evaluation function for calculation and evaluation to determine the drug risk classification based on the PRR method; subsequently, in order to achieve drug risk classification, this study calculated the damage index values of each type of drugs according to the damage index formula and ranked them to determine the risk level of each clustering result, then the number of each type of prescription drugs and over-the-counter drugs, and the proportion of each type of serious. Then, the reliability of the study was initially verified by the number of prescription drugs and over-the-counter drugs and the proportion of each type of serious adverse reactions, and then the signal proportion of the top 10 key adverse reactions was counted in turn; finally, on the basis of the risk classification results and the signal proportion, the pharmacological correlation of each drug class was analysed and evaluated by searching the data for each risk class of drugs to further verify the rationality and feasibility of this experiment.

The article "Regression Analysis of Factors Based on Cluster Analysis of Acute Radiation Pneumonia due to Radiation Therapy for Lung Cancer" was retracted in 2023. Reasons: signs of a paper mill; suspected computer-generated content; unreliable results or conclusions; lack of ethics approval or compliance.

The DB indicator, KL indicator, HS indicator, and the GA indicator proposed in this paper were used to evaluate the validity of the clustering results for these three datasets, and the best number of clusters evaluated by each indicator was used as the criterion to measure the merit of each indicator. The experimental results are shown in Figure 6.

The comparison table of cluster validity indicators in Figure 6 shows that the GA indicator can find the best clusters for these three datasets, while the traditional DB indicator cannot get the accurate clusters for each dataset, and the KL indicator can only find the accurate clusters for the BUPA dataset but cannot find the best clusters for the PID and BCW datasets. In this paper, the criterion for evaluating a cluster validity index is whether the index can accurately find the true class number of the dataset, and if it can find the true class number of the dataset, it means that the cluster validity index is reasonable and effective for evaluating the clustering results. Through the experimental results, it can be proved that the GA index proposed in this paper is more effective and stable than the traditional clustering validity index. The main research direction of this paper is how to determine the optimal number of clusters in cluster analysis scientifically and effectively. Cluster analysis is an important multivariate statistical analysis method, which can help people get the distribution pattern of data when facing the cluttered data, to grasp the intrinsic structure and characteristics of the data set. In the field of big data analysis, including machine learning and pattern recognition, cluster analysis often plays an important role in data analysis as one of the means of data mining, so the study of cluster analysis has great significance.

The article "Regression Analysis of Factors Based on Cluster Analysis of Acute Radiation Pneumonia due to Radiation Therapy for Lung Cancer" was retracted in 2023. Reasons: signs of a paper mill; suspected computer-generated content; unreliable results or conclusions; lack of ethics approval or compliance.

### 4.2. Multifactor Regression Results

The samples in the same cluster have higher similarity, and the samples of different clusters have higher dissimilarities. Although the cluster analysis has a history of decades, the results are obtained due to different clustering methods. The cluster structure has multiple output modes. A multifactorial unconditional logistic regression analysis of the factors associated with acute radiation pneumonia revealed that lower middle lobe lung cancer, history of chronic lung disease, combined diabetes, FEV1 < 2L before chemotherapy, chemotherapy cycles >2 before radiotherapy, simultaneous application of radiotherapy and chemotherapy, total radiotherapy dose >56 Gy, MLD >15 Gy, V5 >40%, V20 > 25%, and V30 > 18% all increased the risk of acute radiation pneumonia, while a history of smoking is a protective factor against the development of acute radiation pneumonia and decreases its risk (all *P* < 0.05, OR < 1), with ORs within the 95% CI interval, as shown in Figure 7.

Smoking is generally considered to be the main risk factor. Smoke is acidic, which tends to make patients form an acidic body, and an acidic body has the risk of inducing lung cancer; environmental pollution also increases the risk of lung cancer; tin, arsenic, and toluene are carcinogenic substances, and air pollution will lead to an increase in these components in the air, thus increasing the risk of lung cancer; chronic lung diseases are also a major risk factor for lung cancer and lung diseases lesions, which can lead to a decrease in lung cell activity and immune capability, increasing the risk of lung cancer; in addition, factors such as occupation and oncogene activation can also increase the risk of lung cancer. The treatment methods of lung cancer include surgery, chemotherapy, and radiotherapy. Surgery is mostly used for the treatment of early-stage tumours, while radiotherapy is the most common treatment method in clinical practice, and according to statistics, more than 60% of lung cancer patients need radiotherapy. Radiotherapy has high clinical value and can effectively improve the local cancer control rate and overall treatment efficiency. The data is preprocessed, and the processed data retains as much information as possible through feature engineering. Select the corresponding clustering algorithm according to the structure of the data; select the appropriate cluster validity index to check the validity of the clustering results. 3D-CRT is the most used radiotherapy treatment for lung cancer in clinical practice. 3D-CRT is based on CT simulation and computer calculation to obtain the real situation of dose distribution, and based on this, the radiotherapy plan is scientifically set to maximize the irradiation of tumour while minimizing the damage to the surrounding tissues and organs. To optimize the clinical effect of radiotherapy implementation, the radiation treatment plan is scientifically set based on the realistic dose distribution based on CT simulation and computer calculation.

The article "Regression Analysis of Factors Based on Cluster Analysis of Acute Radiation Pneumonia due to Radiation Therapy for Lung Cancer" was retracted in 2023. Reasons: signs of a paper mill; suspected computer-generated content; unreliable results or conclusions; lack of ethics approval or compliance.

Because whole lung V20 is an independent influencing factor for grade ≥2 radiation pneumonia, the value of whole lung V20 was entered into the ROC curve, and the area under the whole lung V20 curve was 0.642, as shown in Figure 8. The area under the ROC curve ranges from 0.5 to 1.0, and an area under the ROC curve of 0.5 to 0.7 indicates a low diagnostic value, between 0.7 and 0.9 indicates a moderate diagnostic value, and greater than 0.9 indicates a high diagnostic value. In general, an area under the ROC curve of 0.5–0.7 indicates low diagnostic value, between 0.7 and 0.9 indicates moderate diagnostic value, and above 0.9 indicates high diagnostic value. In the present study, the area under the V20 curve of the whole lung was calculated to be 0.642, which indicates that it has a diagnostic value.

The sensitivity and false-positive rate of whole lung V20 at each point on the ROC curve were used to calculate the value of all cut-off points, and the diagnostic index corresponding to the maximum cut-off value is the optimal diagnostic threshold of 25.9%. When developing a radiation treatment plan, the dosimetry parameters of whole lung V20 are recommended to be limited to ≤25.9%. If this threshold is exceeded, the risk of grade ≥2 radiation pneumonia will increase.

## 5. Conclusion

In this study, we first calculated the damage index values of each drug class according to the damage index formula, and based on this, we ranked to determine the risk level of each clustering result; then we initially verified the reliability of the study with the number of each type of prescription drugs and over-the-counter drugs and the proportion of each type of serious adverse reactions and then counted the signal weight of the top 10 key adverse reactions in turn; finally, based on the risk classification results obtained and the signal weight and based on the results of the risk classification and the proportion of the signal, the pharmacological correlation of each drug class was analysed and evaluated to further verify the rationality and feasibility of this experiment. Therefore, the object will be closer to its centre; however, as the number of clusters increases, the average level of distortion continues to decrease. As the number of clusters increases, the place where the level of distortion decreases the most corresponds to the cluster value is the elbow, and cluster analysis can be performed with the cluster value corresponding to the elbow as the best cluster value. No association was found between gender, age, and the occurrence of grade ≥2 radiation pneumonia in this study. There is no evidence-based medical evidence to confirm that gender and age are the main influencing factors for the occurrence of radiation pneumonia, and in the one-way ANOVA, gender and the occurrence of severe acute radiation pneumonia were not related. The present study did not suggest any guiding indexes in terms of clinical factors. Considering the special situation that about 40% of the patients in this group were hospitalized in sister departments such as surgery or chemotherapy during radiotherapy, the occurrence and classification of radiation pneumonia mainly relied on the medication records and course records of the bedside doctors in different departments; there may be interfering factors other than the existing common clinical factors that we have not yet explored. The next study will be a prospective clinical study to further refine and improve the study of clinical factors in radiation pneumonia.

The article "Regression Analysis of Factors Based on Cluster Analysis of Acute Radiation Pneumonia due to Radiation Therapy for Lung Cancer" was retracted in 2023. Reasons: signs of a paper mill; suspected computer-generated content; unreliable results or conclusions; lack of ethics approval or compliance.

## Figures and Tables

**Figure 1:** Framework of the clustering analysis algorithm.

**Figure 2:** Flow of the algorithm for determining the optimal number of clusters.

**Figure 3:** Comparison of relevant indexes between patients in acute radiation pneumonia group and normal radiotherapy group.

**Figure 4:** Multifactor regression experiment.

**Figure 5:** Summary of data after signal detection and processing.

**Figure 6:** Table of experimental results for comparison of clustering validity indexes.

**Figure 7:** Factorial unconditional logistic regression analysis.

**Figure 8:** ROC curve of the whole lung V20.

## Data Availability

The data used to support the findings of this study are available from the corresponding author upon request.

## References

[1] Bousabarah K., Blanck O., Temming S. (2021). Radiomics for prediction of radiation-induced lung injury and oncologic outcome after robotic stereotactic body radiotherapy of lung cancer: results from two independent institutions. *Radiation Oncology*.

[2] Cui S., Ten Haken R. K., El Naqa I. (2021). Integrating multiomics information in deep learning architectures for joint actuarial outcome prediction in non-small cell lung cancer patients after radiation therapy. *International Journal of Radiation Oncology, Biology, Physics*.

[3] Tinkle C. L., Singh C., Lloyd S. (2021). Stereotactic body radiation therapy for metastatic and recurrent solid tumors in children and young adults. *International Journal of Radiation Oncology, Biology, Physics*.

[4] Siddique S., Chow J. C. L. (2020). Artificial intelligence in radiotherapy. *Reports of Practical Oncology and Radiotherapy*.

[5] Wang J., Liu R., Zhao Y. (2020). A predictive model of radiation-related fibrosis based on the radiomic features of magnetic resonance imaging and computed tomography. *Translational Cancer Research*.

[6] Hess C. B., Nasti T. H., Dhere V. R. (2021). Immunomodulatory low-dose whole-lung radiation for patients with coronavirus disease 2019-related pneumonia. *International Journal of Radiation Oncology, Biology, Physics*.

[7] Nie X., Li L., Yi M. (194). The intestinal microbiota plays as a protective regulator against radiation pneumonitis. *Radiation Research*.

[8] Wang X. S., Shi Q., Mendoza T. (2020). Minocycline reduces chemoradiation-related symptom burden in patients with non-small cell lung cancer: a phase 2 randomized trial. *International Journal of Radiation Oncology, Biology, Physics*.

[9] Pradhan K., Chawla P. (2020). Medical Internet of things using machine learning algorithms for lung cancer detection. *Journal of Management Analytics*.

[10] Tian L., Wang W, Yu B, Zhang G (2020). Efficacy of dendritic cell-cytokine induced killer cells combined with concurrent chemoradiotherapy on locally advanced non-small cell lung cancer. *Journal of B.U.ON.: Official Journal of the Balkan Union of Oncology*.

[11] Quirk M. T., Lee S., Murali N., Genshaft S., Abtin F., Suh R. (2020). Alternatives to surgery for early-stage non-small cell lung cancer. *Clinics in Chest Medicine*.

[12] Fouillade C., Curras-Alonso S., Giuranno L. (2020). FLASH irradiation spares lung progenitor cells and limits the incidence of radio-induced senescence. *Clinical Cancer Research*.

[13] Vogelius I. R., Petersen J., Bentzen S. M. (2020). Harnessing data science to advance radiation oncology. *Molecular oncology*.

The article "Regression Analysis of Factors Based on Cluster Analysis of Acute Radiation Pneumonia due to Radiation Therapy for Lung Cancer" was retracted in 2023. Reasons: signs of a paper mill; suspected computer-generated content; unreliable results or conclusions; lack of ethics approval or compliance.

[14] Kim H., Hong H., Yoon S. H. (2020). Diagnostic performance of CT and reverse transcriptase polymerase chain reaction for coronavirus disease 2019: a meta-analysis. *Radiology*.

[15] Travis W. D., Dacic S., Wistuba I. (2020). IASLC multidisciplinary recommendations for pathologic assessment of lung cancer resection specimens after neoadjuvant therapy. *Journal of Thoracic Oncology*.

[16] Martini K., Baessler B., Bogowicz M. (2021). Applicability of radiomics in interstitial lung disease associated with systemic sclerosis: proof of concept. *European Radiology*.

[17] Kim J. W., Park E. Y. (2020). Self-management of oxygen and bronchodilators to relieve the dyspnoea of lung cancer with pneumoconiosis. *International Journal of Palliative Nursing*.

[18] Kurz C. F., Stafford S. (2020). Isolating cost drivers in interstitial lung disease treatment using nonparametric Bayesian methods. *Biometrical Journal*.

[19] Bolourani S., Tayebi M. A., Diao L. (2021). Using machine learning to predict early readmission following esophagectomy. *The Journal of Thoracic and Cardiovascular Surgery*.

[20] Kaneko H., Itoh H., Yotsumoto H. (2020). Association of cancer with outcomes in patients hospitalized for heart failure. *Circulation Journal*.

